# Elucidating the Mechanism of Action of Salvia miltiorrhiza for the Treatment of Acute Pancreatitis Based on Network Pharmacology and Molecular Docking Technology

**DOI:** 10.1155/2021/8323661

**Published:** 2021-11-24

**Authors:** Kunyao Zhu, Man Zhang, Jia Long, Shuqi Zhang, Huali Luo

**Affiliations:** ^1^Clinical College of Chongqing Medical University, Chongqing 401331, China; ^2^College of Traditional Chinese Medicine, Chongqing Medical University, Chongqing 401331, China; ^3^Chongqing Key Laboratory of Traditional Chinese Medicine for Prevention and Cure of Metabolic Diseases, Chongqing Medical University, No. 1 Yixueyuan Road, Yuan Jiagang, Yuzhong District, Chongqing 400016, China

## Abstract

Using network pharmacology and molecular docking, this study investigated the molecular mechanisms by which the active components in *Salvia miltiorrhiza* can alleviate acute pancreatitis. Initially, the active components of *Salvia miltiorrhiza* and the targets collected from the GeneCards database were screened based on the platform of systematic pharmacology analysis of traditional Chinese medicine. Subsequently, the active components were intersected with the disease targets. Also, interactions among the targets were computed using the STRING database. Biological function and pathway enrichment were analyzed using the Cluster Profiler package in the R software. Protein-protein interaction and component target pathway network were constructed using the Cytoscape software. Ultimately, the key targets and their corresponding components in the network were verified using the AutoDock Vina software. The results showed *Salvia miltiorrhiza* had 111 targets for acute pancreatitis. The biological process (BP) analysis showed that the active components of *Salvia miltiorrhiza* induced a drug response, positive regulation of transcription by RNA polymerase II promoter, signal transduction, positive regulation of cell proliferation, and negative regulation of apoptosis. Furthermore, the KEGG enrichment analysis screened 118 (*P* < 0.05) signaling pathways, such as the pathways related to cancer, neuroactive ligand-receptor interaction, PI3K-Akt signaling pathway, and cAMP signaling pathway, to name a few. Finally, molecular docking showed that the active components of *Salvia miltiorrhiza* had a good binding affinity with their corresponding target proteins. Through network pharmacology, this study predicted the potential pharmacodynamic material basis and the mechanisms by which *Salvia miltiorrhiza* can treat acute pancreatitis. Moreover, this study provided a scientific basis for mining the pharmacodynamic components of *Salvia miltiorrhiza* and expanding the scope of its clinical use.

## 1. Introduction

Acute pancreatitis (AP) is a common clinical inflammatory disease caused by the abnormal activation of trypsinogen. Approximately 15-25% of the patients with this abnormality might develop severe acute pancreatitis. Also, clinical treatment of AP is difficult for several reasons, including the rapid development of the disease, many complications, and high mortality. Therefore, it is necessary to find a cure for AP. *Salvia miltiorrhiza*, an inexpensive and easily available traditional medicine, may be used as a routine drug in the comprehensive treatment of AP. It promotes blood circulation, removes blood stasis, dredges channels, relieves pain, dilates microvessels, and improves microcirculation. Clinical studies reported the significant role of [1] *Salvia miltiorrhiza* in the treatment of AP. However, the specific mechanism by which *Salvia miltiorrhiza* can alleviate AP is unclear. Further studies are required to identify the specific disease targets of the components of *Salvia miltiorrhiza*.

Network pharmacology has recently become popular globally. It provides a holistic perspective of the relationship between drugs and diseases by constructing a “drug-gene target disease” network. Due to its holistic and systematic characteristics, it has been widely used to predict the potentially active components in traditional Chinese medicine and study their mechanism of action on disease targets.

Molecular docking, an essential method of virtual drug screening, is important for modern pharmacological research. It predicts the binding affinity between drugs and receptors by computing the interactions and binding energy between small-molecule ligands (drugs) and protein receptors. This study used a combination of network pharmacology and molecular docking methods to investigate the mechanism of action of the active components of *Salvia miltiorrhiza* for the treatment of acute pancreatitis. It provides a theoretical basis for the screening of the active components of *Salvia miltiorrhiza* and promotes further research on *Salvia miltiorrhiza*.

## 2. Materials

The database, analysis platform, and software used in this study are shown in Table 1.

## 3. Methodology

### 3.1. Construction and Screening of Chemical Constituents of *Salvia miltiorrhiza* Bge

We used the Chinese medicine systems pharmacology analysis platform TCMSP and inserted “Danshen” as the keyword to retrieve all its chemical components. Pharmacokinetics (oral bioavailability) and drug-like (DL) are often used by researchers to screen for active ingredients. OB values indicate the percentage of drugs that enter the human circulation. High OB values are usually the key indicators for evaluating the effectiveness of drugs. DL values indicate the degree of similarity between the components of traditional Chinese medicine and known chemical drugs. It is important for determining whether the components of Chinese Materia medica can exhibit pharmacological activities in organisms.

Drug-likeness (DL) is based on the analysis of the physicochemical properties and/or structural characteristics of existing small organic drugs, especially those with undesirable properties, for example, compounds with poor ADMET (absorption, distribution, metabolism, excretion, and toxicity) [2]. Based on the molecular descriptors and the Tanimoto coefficients, the research team of RU [3] and others constructed a model to evaluate DL in the TCMSP database represented as *T*(*A*, *B*) = *A* · *B*/‖*A*‖^2^ + ‖*B*‖^2^ − *A* · *B*, where *A* is the molecular descriptor for a given herbal component, and *B* represents the average value of this property for all molecules in the drug bank database [4].

DL is related to simple molecular properties such as molecular weight, physicochemical properties, and the number of convertible bonds or aromatic rings. In general, DL is related to the potential success of drug discovery in terms of pharmacokinetics and safety [5]. Because the discovery of drugs from candidate compounds is not always successful, the DL method has been widely used to screen compounds with undesirable properties, especially those with poor ADMET spectra. For TCPSP database compounds, DL ≥ 0.18 has been used as a standard for screening bioactive compounds through the traditional Chinese medicine systems pharmacology analysis [3, 4].

In conclusion, the active components of *Salvia miltiorrhiza* were screened under the conditions of OB ≥ 30% and DL ≥ 0.18, and the information of the qualified compounds was recorded and maintained in a tabular form using Microsoft Excel. Additionally, the quality control components of *Salvia miltiorrhiza* and the reported compounds with definite biological activities in the Chinese Pharmacopoeia were also analyzed as candidates. Then, the chemical structure of the above candidate components was constructed by the ChemBioDraw Ultra software and stored in MOL2 format.

### 3.2. Collection of *Salvia miltiorrhiza* Related Targets

The final list of components was prepared after removing the duplicate active components. This list was used to search the TCMSP analysis platform for targets corresponding to the active components. Furthermore, the gene names of all the targets were obtained using the UniProt database.

### 3.3. Target Acquisition of Acute Pancreatitis

With “acute pancreatitis” as the keyword and the screening criterion set as median screening, disease-related targets were retrieved using the GeneCards database. “Median screening” ensured the reliability of the candidate targets. Furthermore, the names of AP-related targets were standardized using the UniProt database.

### 3.4. Screening of Common Drug-Disease Targets and Construction of the PPI Network

Venny 2.1 was used to build a Wayne map by providing *Salvia miltiorrhiza* and AP as the component target and disease target, respectively. The map provided information about common targets. These common targets were imported into the STRING database after specifying the “species” and “minimum required interaction score” as “Homo sapiens” and “≥0.99,” respectively. The resultant protein interaction (PPI) information was imported into the Cytoscape software for topological analysis and construction of the PPI network diagram.

### 3.5. Gene Enrichment Analysis

The function of these common targets in signal pathways was further investigated using the GO function and KEGG pathway enrichment (*P* < 0.05), which were in turn computed using the Cluster Profiler package in the R software.

### 3.6. Network Construction

Data comprising the active components and their corresponding targets were stored in files and imported to the Cytoscape software, where the component-target network diagram was constructed. This network was used to investigate the pharmacological mechanism of action of the active components of *Salvia miltiorrhiza*. Furthermore, the components and their AP targets underwent reverse screening based on the first 20 pathways enriched by KEGG. Subsequently, these screened data were used to build a network relation table of “components-targets-pathways” using the Cytoscape software.

### 3.7. Core Components and Targets of Molecular Docking Verification

From the constructed “Component-Target-Pathway” network, the components and their corresponding targets with moderate to high values were selected for molecular docking studies using AutoDock Vina. A series of steps were performed during molecular docking. (i) The 3D structure of the target protein was retrieved from the PDB database, and the ligand and nonprotein molecules (such as water molecules) were removed using the PyMoL software. The target protein files were saved in the PDB format. (ii) The target protein and the components of *Salvia miltiorrhiza* (in mol2 format) were converted into the pdbqt file format. (iii) The active site in the target protein was prepared for docking by setting the proper Grid Box size and coordinates. Then, the active components of *Salvia miltiorrhiza* were docked to the active site of the target protein. (iv) Finally, the components that demonstrated the lowest binding energy and highest binding affinity toward the target proteins were selected. The docked complexes of the selected components were visualized using the PyMoL software.

## 4. Results

### 4.1. Screening for the Active Components of *Salvia miltiorrhiza*

A total of 202 active chemical components of *Salvia miltiorrhiza* were retrieved in this study. Using specific screening criteria, such as OB ≥ 30%, DL ≥ 0.18, searching for quality control components in the Chinese Pharmacopoeia, and the removal of nontarget components, 65 active components of *Salvia miltiorrhiza* were selected. These components are presented in Table 2.

### 4.2. Screening of Target Compounds in *Salvia miltiorrhiza* Bunge

From the TCPSP database, 65 candidate targets of *Salvia miltiorrhiza* were selected. After removing the inactive components, 58 active components of *Salvia miltiorrhiza* Bunge were selected, and their corresponding 919 targets were obtained. Finally, the gene names corresponding to the target protein names were obtained from the UniProt database.

### 4.3. Component-Target Network Analysis of *Salvia miltiorrhiza* Bunge

As shown in Figure 1, the DANSHEN component-target network contained 173 nodes (58 candidate components and 115 associated targets) and 744 edges. Network topology analysis was performed using the network analyzer function in Cytoscape. The degree value (degree) is an important index for describing network nodes. The average number of target sites per compound was 12.83, and the average number of target sites per compound was 6.47. It was found that 14 targets interacted with ≥20 active compounds. The top 10 compounds were luteolin (Mol000006), tanshinone IIA (Mol007154), dihydrotanshinolactone (Mol007100), tanshinone D (Mol007093), 4-methyltanshinone (Mol007049), salvianol ketone (Mol007145), isocyantanshinone (Mol007108), 2-isopropyl-8-methylphenanthrene-3,4-dione (Mol007041), neocryptotanshinone II (Mol007124), and tanshinone I (Mol007119). Additionally, more than 25 targets interacted with ≥10 active compounds. The top 10 targets were PTGS2, NCOA1, SCN5A, OPRM1, CHRM1, ADRB2, F2, CA2, CHRNA7, and ACHE. The results suggested that a single component of *Salvia miltiorrhiza* affected multiple targets.

### 4.4. Target Screening and PPI Network Analysis of *Salvia miltiorrhiza* in Treatment of Acute Pancreatitis

Using “acute pancreatitis” as the keyword, 8,319 targets were obtained from the Genecards database. After the median screening of these targets, 4,167 targets were selected. Later, the interaction of 145 active components of *Salvia miltiorrhiza* with the 4,167 targets related to acute pancreatitis was investigated, and 111 common targets were found. These results indicated the active role of the components of *Salvia miltiorrhiza* in acute pancreatitis through their interaction with multiple targets (Figure 2).

### 4.5. Analysis of Target-Protein Interaction Network

To further investigate the mechanism of interaction between the components of *Salvia miltiorrhiza* and the targets of AP, the 111 common targets were introduced into the STRING database for PPI network analysis (Figure 3). The results of this analysis were imported into Cytoscape 3.8.0 to construct the PPI network. There were 54 nodes and 82 edges in the PPI network, and the average degree of freedom was 9.13. In the PPI network, 65 protein degrees were higher than the average, and eight key nodes had moderate values according to their target nodes. These eight nodes, viz., PTGS2, NCOA1, SCN5A, OPRM1, CHRM1, ADRB2, F2, and PTGS1, were selected for further analysis. The proteins indicated by these key nodes interacted with a higher number of target proteins compared to the proteins in the other nodes in the PPI network. Hence, these nodes played an important role in the PPI network.

### 4.6. GO Function and KEGG Pathway Enrichment Analysis

In the GO enrichment analysis, 503 biological processes (defined as a series of events generated by an orderly combination of one or more molecular functions, BP), 113 molecular functions (described as activity at the molecular level, MF), and 59 cell components (each part of the cell and extracellular environment, CC) were obtained. The resultant BP, MF, and CC were sorted according to corrected *P* values. Then, to better describe the statistical significance of the conclusion data, the top 20 BP, MF, and CC were used to draw bubble charts and histograms, as shown in Figures 4–11. In the bubble chart, the size of the bubble represented the number of genes enriched in BP, CC, and MF entries, while different bubble colors represented different enrichment degrees of target genes in each BP, CC, and MF entry. From the results of the GO analysis, it was observed that many BP, with a high enrichment degree and a large number of enriched genes, were mainly involved in drug response, positive regulation of RNA polymerase, promoter transcription, signal transduction, positive regulation of cell proliferation, and negative regulation of apoptosis. Additionally, 118 signaling pathways (*P* < 0.05), screened using KEGG enrichment analysis, mainly involved pathways related to cancer, neuroactive ligand-receptor interaction signaling pathway, PI3K-Akt signaling pathway, and cAMP signaling pathway (Table 3).

### 4.7. Analysis of “Composition-Target-Pathway” Network of *Salvia miltiorrhiza*

From the KEGG enrichment analysis, the top 20 pathways with 153 targets for AP and 58 active ingredients of *Salvia miltiorrhiza* were selected. A “component-target-pathway” was constructed with the selected targets and compounds using the Cytoscape software (Figure 12). Among the compounds, luteolin, tanshinone IIA, dihydrodanshen lactone, 2-isopropyl-8-methylphenyl-3, 4-dione, 4-methyltanshinone, and tanshinone had the highest values. Among the targets, the highest values were displayed by PTGS2, NCOA1, CHRM1, and OPRM1. The compounds and targets with the highest values in the network were the most effective for the treatment of acute pancreatitis. Also, the components of *Salvia miltiorrhiza* could resist pancreatitis injury through a multicomponent multitarget-multipathway.

### 4.8. Molecular Docking Verification of the Key Target of *Salvia miltiorrhiza*

A previous study reported that the stability of the binding conformation of the target protein with the ligand (active component) depends on the binding energy of the docked complex such that the lower binding energy of the docked complex increases the stability of the binding conformation. Binding energies of ≤-4.25 kcal/mol, ≤-5.0 kcal/mol, and ≤ -7.0 kcal/mol indicated reasonable binding affinity, good binding affinity, and strong binding affinity, respectively. To confirm the results of the network analysis, four targets with high median scores from the “component-target-pathway,” which included PTGS2, RELA, TNF, and AKT1, were selected as receptors for molecular docking studies. Six active components of *Salvia miltiorrhiza*, designated as the six core components, were used as ligands for docking analysis using AutoDock Vina. The docking results are shown in Table 4. All the six core components of *Salvia miltiorrhiza*-*Paleonia vulgaris* showed binding energies of ≤-5 kcal/mol with the receptors (target proteins). It was observed that 83.3% of the components had binding energies ≤–7.5 kcal/mol with their targets. This indicated a strong binding affinity of the components of *Salvia miltiorrhiza*-*Paleonia vulgaris* with the target proteins. The binding affinities of the components of *Salvia miltiorrhiza* including new quinone D and tanshinone IIA to receptor-PTGS2 and the components such as Salviol ketone and quercetin to receptor-OPRM1 were higher than the binding affinity between these receptors and their original ligands. Additionally, the docking results confirmed the reliability of the results of network pharmacological analysis (Table 4). Finally, the PyMoL software was used to visualize the docked complexes. The docked complexes with low binding energies are illustrated in Figure 13.

## 5. Conclusion

TCM deems that inflammation of internal organs may be due to accumulation of pathogenic qi, dampness, and heat. Qi stagnation causes blood stasis, and dampness leads to distention. When the pathogenic heat flames extremely, carbuncle will form. Acute pancreatitis is classified into “abdominal pain” or “internal carbuncle” in TCM. It can be relieved by the treating principles as follows: promoting qi and blood circulation and removing pathogenic heat by purgation [6].

In this study, the best tanshinones and flavonoid were screened from the high-frequency danshen which was used to treat AP by TCPSP and PubChem database, it is suggested that tanshinones and flavones in Salvia miltiorrhiza may be the main material basis for the treatment of AP. The former includes tanshinone iia, 4-methylenemiltirone, salviolone, neocryptotanshinone ii, and isocryptotanshi-none, and the latter includes luteolin. To further identify the key compounds of Salvia miltiorrhiza in the treatment of AP, we constructed a composite target network, and the compounds in the top 10 degrees were luteolin, tanshinone iia, dihydrotanshinolide, dan-shexinkum d,4-methylenemiltirone salviolone, isocryptotanshi-none, 2-isopropyl-8-methylphenanthrene-3,4-dione, neocryptotanshinone ii, and miltionone I.

It was found that [7] luteolin protected SAP mice by inducing ho-1-mediated anti-inflammatory and antioxidant activities and inhibiting the activation of the NF-*Κ*B pathway, which demonstrated that luteolin could significantly improve the infiltration and necrosis of inflammatory cells in the pancreas. A study by Chen et al. [8] confirmed that tanshinone IIA can inhibit oxidative stress through the NRF2ROS pathway and protect mice from acute pancreatitis. Isocryptotanshinone is a tanshinone monomer, which is the active component of *Salvia miltiorrhiza*. Antibacterial, anti-inflammatory, blood stasis promoting, wound healing, and other effects can play a positive therapeutic role in all aspects of the treatment of AP [9]. In conclusion, several key compounds in *Salvia miltiorrhiza* can not only inhibit the release of inflammatory factors and reduce the inflammatory reaction but also reduce the absorption of intestinal endotoxin and the translocation of pathogenic bacteria. They can also inhibit the growth of cancer cells and play an important role in improving microcirculation and alleviate edema and necrosis of pancreatic tissue. Many studies [10, 11] have shown that neocryptotanshinone, which is a diterpenoid isolated from *Salvia miltiorrhiza*, can inhibit LPS-induced inflammation by inhibiting NF-*κ*B and iNOS signals. In a study by Fan et al. [12], it was found that neocryptotanshinone II, a monomer found in *Salvia miltiorrhiza*, plays an important role in the regulation of inflammatory cytokines and their signal pathways. TNF, IL-6, and NFKB1 are involved in the inflammation-related pathways, such as the IL-17 signal pathway and the TNF signal pathway, to regulate the inflammatory response in the body.

The composition-target network of Radix *Salvia miltiorrhiza* reflects its anti-inflammatory and anti-injury characteristics. Based on network analysis, PTGS2, NCOA1, SCN5A, OPRM1, CHRM1, ADRB2, CHRNA7, and ACHE were selected as the key targets of AP.

Studies [13] have shown that PTGS2 has an anti-inflammatory effect on AP. NCOA1 can regulate IL-17, participate in the acute inflammatory process of AP, and play an important role in autoimmunity [14]. It has been reported [15] that tanshinone IIA, an active component of *Salvia miltiorrhiza*, can relieve the mechanical and thermal pain induced by Freund's complete adjuvant by inhibiting the expression of p-ERK and NF-*κ*B. The levels of PTGS2 can reduce inflammation by reducing the levels and mRNA expression of IL-1*β*, IL-6, and tumor necrosis factor in sercytokines IL-1 *β*, IL-6, and TNF-*α*, and hence, can reduce pain. OPRM1 is an opioid receptor. The mu-opioid receptor (MOR) encoded by the OPRM1 gene is the main target of most opioid drugs. It is also an important factor that exerts analgesic effects, imparts tolerance, and provides dependence [16]. Tanshinone IIA might exert an analgesic effect through the action of OPRM1 on the inflammatory sites of the central nervous system and pancreas. CHRM1 might reduce inflammation and disease activity in various animal models of intestinal inflammation through cholinergic activation mechanisms involving the activation of the +7 NACHR subtype [17]. There is growing evidence [18, 19] from AP patients for the existence of cholinergic anti-inflammatory pathways that are completed by the efferent Vagus nerve fibers and are thus able to respond quickly and effectively to the inflammatory state. The results showed [20] that *Salvia miltiorrhiza* can dilate blood vessels, promote blood circulation, and remove blood stasis, and thus, inhibit platelet aggregation, anticoagulation, antithrombus, and reduce plasma viscosity. At the onset of AP, the body experiences increased activation of the sympathetic nervous system, which is marked by an increase in the heart rate and blood pressure. The sympathetic nervous system acts on the *β*1 and *β*2 receptors in the heart and blood vessels, respectively, regulating blood pressure. The ADRB2 gene regulates blood pressure [21], and the *β*2 adrenergic receptor (*β*2-AR), expressed by ADRB2, is extensively present in immune cells. In mice and humans, stimulation of *β*2 AR activates NOD2 signaling, promotes T cell differentiation, and regulates the secretion of related cytokines and inflammation, according to a study [22] on dendritic cells. CHRNA7 regulates the function of immune cells in the spleen and is involved in regulating the production of proinflammatory cytokines, which are an integral part of the cholinergic anti-inflammatory pathway that regulates inflammation [23]. The mechanism by which *Salvia miltiorrhiza* plays an anti-inflammatory role through the cholinergic anti-inflammatory pathway is not clear. By analyzing the KEGG pathway in this study, the authors speculate that CHRNA7 might be expressed in acute pancreatitis and play a key role in regulating inflammation. *Salvia miltiorrhiza* might play an anti-inflammatory role in the cholinergic anti-inflammatory pathway, which might elucidate the anti-inflammatory mechanisms and suggest clinical applications of *Salvia miltiorrhiza*. ACHE, a substance released by cholinergic neurons, is a major transmitter of the parasympathetic nervous system that rapidly hydrolyzes the neurotransmitter acetylcholine ACHE and acts as a marker of systemic inflammation. Clinical studies [24] have shown that a decrease in the serum cholinesterase level is related to the severity of the condition in patients, and a greater decrease indicates higher mortality. Serum cholinesterase levels also drop when the pancreas is severely damaged. Sheng et al. [25] found that serum cholinesterase concentration was an independent risk factor for the prognosis of acute pancreatitis.

Acute pancreatitis is a complicated, acute, and severe disease of the abdomen, with many complications and high mortality, involving different metabolic pathways. The compounds in *Salvia miltiorrhiza* were extracted from the database. The potential targets of *Salvia miltiorrhiza* were predicted among these compounds, and the KEGG pathway enrichment analysis was performed. The potential pathway of *Salvia miltiorrhiza* was obtained based on these targets. According to the KEGG enrichment analysis of the key targets and associated studies, the acute pancreatitis pathway of *Salvia miltiorrhiza* is mainly involved in the PI3K-Akt signaling pathway, HIF-1 signaling pathway, cAMP signaling pathway, cholinergic synapse, FOXO signaling pathway, insulin resistance, AMPK signaling pathway, pathways associated with cancer, pancreatic cancer, neuroactive ligand-receptor interaction, etc.

As an important signal transduction pathway, PI3K/AKT controls a variety of signal transduction pathways, including proliferation, apoptosis, and stress. In the AP model induced by ligation of the pancreatic duct, the expression of p-Akt and the activity of NF-*κ*B in pancreatic tissue were significantly increased [26]. The expression of hypoxia-inducible factor-l*α* (hypoxia-inducible factors-1 *α*, HIF-1 *α*), Beclin1 gene, and microtubule-associated protein-1 light chain 3-II (microtubule-associated protein 1 light chain 3-II, LC3-II) are closely related to the pathological development of inflammation [27–29]. Ischemia, hypoxia, and autophagy are the main characteristics of acute pancreatitis cell injury. HIF-1*α* is very sensitive to the concentration of oxygen in cells and reflects the degree of hypoxia in cells. Inflammatory injury increases the expression of HIF-1*α* and the release of Beclin1 and LC3-II, which are markers of autophagic activity; it also increases the level of autophagy. In pancreatitis, autophagy is activated but lysosomal degradation is inhibited, and the imbalance between increased autophagy and decreased lysosomal degradation leads to autophagy flux arrest, which can cause severe acinar cell degeneration and trypsinogen activation, leading to the development of AP [30]. At the onset of AP, the acute inflammatory response of AP activates the insulin resistance pathway, triggering inflammation and immune responses. Studies [31] have shown that tanshinone monomers (such as tanshinone IIA and cryptotanshinone) can effectively increase glucose consumption, improve insulin resistance, and decrease the activity of the insulin pathway in insulin-resistant cells, which attenuates the inflammatory response and reduces the oxidative stress response in the cell. The cAMP/PKA signaling pathway plays a role in regulating oxidative stress and inflammatory response in AP. Yang et al. [32] showed that inhibition of NF-*κ*b, which is dependent on estrogen receptor *α*, inhibits the production of IL-6, and thus, reduces inflammation. Saito et al. [33] showed that cholinergic synapses can induce an immune-inflammatory response that can cause pancreatic edema and bleeding. The FOXO1 signaling pathway plays an important role in cell metabolism, oxidative stress, cell proliferation, and apoptosis [34]. The oxidative stress response induced by AP can target the insulin signaling pathway via the FOXO signaling pathway to maintain homeostasis and mitigate tissue damage. Imbalance in the AMPK signal pathway is closely related to oxidative stress [35–38]. The mechanism of action of *Salvia miltiorrhiza* Bunge on the AMPK signal pathway is not clear; however, the authors speculate that *Salvia miltiorrhiza* Bunge might increase the activity of AMPK, decrease the level of ROS, increase the production of SOD, and enhance the antioxidative ability of an organism. The reduction of oxidative stress in acute pancreatitis might provide important directions for the study of the mechanism of oxidative stress and clinical application of *Salvia miltiorrhiza*.

In summary, using network pharmacology methods and molecular docking techniques, this study identified quercetin and other active components in *Salvia miltiorrhiza* to be effective against acute pancreatitis by targeting PTGS2, NCOA1, and other key genes. The results of the KEGG enrichment analysis indicated that *Salvia miltiorrhiza* might alleviate AP by regulating the PI3K-AKT signal pathway and other signal pathways. This study showed that *Salvia miltiorrhiza* probably affects AP through multiple targets and pathways. In this study, the possible pharmacodynamic basis and the mechanism of action of *Salvia miltiorrhiza* in treating acute pancreatitis were predicted by network pharmacology. The results of molecular docking also showed that the active molecule of *Salvia miltiorrhiza* has good binding activity with key target proteins. This study provides a scientific basis for further experimental research and clinical application.

## Figures and Tables

**Figure 1:** The component-target network of SM.

**Figure 2:** Venn map of “Danshen” target and acute pancreatitis target. Note: the blue part represents the target genes of acute pancreatitis, the red part represents the target genes of the active components of *Salvia miltiorrhiza* to be modified, and the intersection represents the common target genes.

**Figure 3:** The analysis diagram of target-protein interaction network.

**Figure 4:** GO functional enrichment analysis: Bubble diagram of the analysis of the biological processes.

**Figure 5:** GO functional enrichment analysis: Bubble diagram of the analysis of the cell components.

**Figure 6:** GO functional enrichment analysis: Bubble diagram of the analysis of the molecular functions.

**Figure 7:** GO functional enrichment analysis: histogram of the analysis of the biological processes.

**Figure 8:** GO functional enrichment analysis: cellular components analysis.

**Figure 9:** GO functional enrichment analysis: histogram of the analysis of the molecular functions.

**Figure 10:** Bubble diagram of the KEGG pathway enrichment analysis.

**Figure 11:** Histogram of the KEGG pathway enrichment analysis.

**Figure 12:** Component-target pathway network of *Salvia miltiorrhiza.*

**Figure 13:** Schematic diagram of molecular docking between core components of *Salvia miltiorrhiza* and key targets. Note: (a)–(d) are molecular docking diagrams of *Salvia miltiorrhiza* new quinone D and PTGS2, *Salvia miltiorrhiza* new quinone D and CHRM1, tanshinone IIA and NCOA1, and tanshinone IIA and OPRM1, respectively.

**Table 1:** Information of the databases, analysis platform, and software.

Name	Website	Version
TCMSP	http://lsp.nswuaf.edu.cn/tcmsp.php	/
UniProt	http://http//www.uniprot.org	/
GeneCards	http://http//www.genecards.org/	/
STRING	http://http//string-db.org/	/
Cytoscape	http://cytoscape.org/	3.8.0
Venny	http://biofogp.cnb.csic.es/tools/venny	/
DAVID	http://david.ncifcrf.gov/	/
R-project	https://www.r-project.org/	4.0.3
PDB	https://www.rcsb.org/	/
MGLTools	http://mgltools.scripps.edu/	1.5.6
PyMoL	https://pymol.org/2/	1.7.2.1
AutoDock Vina	http://vina.scripps.edu/	1.1.2

**Table 2:** Information of the candidate components of *Salvia miltiorrhiza.*

	MOl ID	Molecule Name	OB(%)	DL	Herb
1	MOL001601	1,2,5,6-tetrahydrotanshinone	38.75	0.36	SM
2	MOL001659	Poriferasterol	43.83	0.76	SM
3	MOL001771	poriferast-5-en-3beta-ol	36.91	0.75	SM
4	MOL001942	isoimperatorin	45.46	0.23	SM
5	MOL002222	sugiol	36.11	0.28	SM
6	MOL002651	Dehydrotanshinone II A	43.76	0.4	SM
7	MOL002776	Baicalin	40.12	0.75	SM
8	MOL000569	digallate	61.85	0.26	SM
9	MOL000006	luteolin	36.16	0.25	SM
10	MOL006824	*α*-amyrin	39.51	0.76	SM
11	MOL007036	5,6-dihydroxy-7-isopropyl-1,1-dimethyl-2,3-dihydrophenanthren-4-one	33.77	0.29	SM
12	MOL007041	2-isopropyl-8-methylphenanthrene-3,4-dione	40.86	0.23	SM
13	MOL007045	3*α*-hydroxytanshinoneIIa	44.93	0.44	SM
14	MOL007048	(E)-3-[2-(3,4-dihydroxyphenyl)-7-hydroxy-benzofuran-4-yl]acrylic acid	48.24	0.31	SM
15	MOL007049	4-methylenemiltirone	34.35	0.23	SM
16	MOL007050	2-(4-hydroxy-3-methoxyphenyl)-5-(3-hydroxypropyl)-7-methoxy-3-benzofurancarboxaldehyde	62.78	0.4	SM
17	MOL007051	6-o-syringyl-8-o-acetyl shanzhiside methyl ester	46.69	0.71	SM
18	MOL007058	formyltanshinone	73.44	0.42	SM
19	MOL007059	2-beta-Hydroxymethyllenetanshiquinone	32.16	0.41	SM
20	MOL007061	Methylenetanshinquinone	37.07	0.36	SM
21	MOL007063	przewalskin a	37.11	0.65	SM
22	MOL007064	przewalskin b	110.32	0.44	SM
23	MOL007068	Przewaquinone B	62.24	0.41	SM
24	MOL007069	przewaquinone c	55.74	0.4	SM
25	MOL007070	(6S,7R)-6,7-dihydroxy-1,6-dimethyl-8,9-dihydro-7H-naphtho[8,7-g]benzofuran-10,11-dione	41.31	0.45	SM
26	MOL007071	przewaquinone f	40.31	0.46	SM
27	MOL007077	sclareol	43.67	0.21	SM
28	MOL007079	tanshinaldehyde	52.47	0.45	SM
29	MOL007081	Danshenol B	57.95	0.56	SM
30	MOL007082	Danshenol A	56.97	0.52	SM
31	MOL007085	Salvilenone	30.38	0.38	SM
32	MOL007088	cryptotanshinone	52.34	0.4	SM
33	MOL007093	dan-shexinkum d	38.88	0.55	SM
34	MOL007094	danshenspiroketallactone	50.43	0.31	SM
35	MOL007098	deoxyneocryptotanshinone	49.4	0.29	SM
36	MOL007100	dihydrotanshinlactone	38.68	0.32	SM
37	MOL007101	dihydrotanshinoneI	45.04	0.36	SM
38	MOL007105	epidanshenspiroketallactone	68.27	0.31	SM
39	MOL007107	C09092	36.07	0.25	SM
40	MOL007108	isocryptotanshi-none	54.98	0.39	SM
41	MOL007111	Isotanshinone II	49.92	0.4	SM
42	MOL007115	manool	45.04	0.2	SM
43	MOL007118	microstegiol	39.61	0.28	SM
44	MOL007119	miltionone I	49.68	0.32	SM
45	MOL007120	miltionone II	71.03	0.44	SM
46	MOL007121	miltipolone	36.56	0.37	SM
47	MOL007122	Miltirone	38.76	0.25	SM
48	MOL007123	miltirone II	44.95	0.24	SM
49	MOL007124	neocryptotanshinone ii	39.46	0.23	SM
50	MOL007125	neocryptotanshinone	52.49	0.32	SM
51	MOL007127	1-methyl-8,9-dihydro-7H-naphtho[5,6-g]benzofuran-6,10,11-trione	34.72	0.37	SM
52	MOL007130	prolithospermic acid	64.37	0.31	SM
53	MOL007132	(2R)-3-(3,4-dihydroxyphenyl)-2-[(Z)-3-(3,4-dihydroxyphenyl)acryloyl]oxy-propionic acid	109.38	0.35	SM
54	MOL007140	(Z)-3-[2-[(E)-2-(3,4-dihydroxyphenyl)vinyl]-3,4-dihydroxy-phenyl]acrylic acid	88.54	0.26	SM
55	MOL007141	salvianolic acid g	45.56	0.61	SM
56	MOL007142	salvianolic acid j	43.38	0.72	SM
57	MOL007143	salvilenone I	32.43	0.23	SM
58	MOL007145	salviolone	31.72	0.24	SM
59	MOL007149	NSC 122421	34.49	0.28	SM
60	MOL007150	(6S)-6-hydroxy-1-methyl-6-methylol-8,9-dihydro-7H-naphtho[8,7-g]benzofuran-10,11-quinone	75.39	0.46	SM
61	MOL007151	Tanshindiol B	42.67	0.45	SM
62	MOL007152	Przewaquinone E	42.85	0.45	SM
63	MOL007154	tanshinone iia	49.89	0.4	SM
64	MOL007155	(6S)-6-(hydroxymethyl)-1,6-dimethyl-8,9-dihydro-7H-naphtho[8,7-g]benzofuran-10,11-dione	65.26	0.45	SM
65	MOL007156	tanshinone VI	45.64	0.3	SM

**Table 3:** The information of the top 20 pathways in the KEGG pathway enrichment analysis.

No.	Pathway	Gene	*P* value	Gene count
1	hsa05200: pathways in cancer	RB1, GSK3B, CDKN1A, GSTP1, PTGS2, ADCY8, RELA, EGFR, PIK3CG, CASP9, EDNRA, RXRA, CCND1, MYC, CASP3, ERBB2, AKT1, MAPK1, PRKACA, JUN, HSP90AA1, NOS2, MMP1, MMP2, STAT3, FOS, MMP9, VEGFA, NFKBIA, AR, IL6, CDK4, CDK2, BCL2, MDM2, BIRC5, PPARG, MET, TP53, BCL2L1	7.57E-20	44
2	hsa04080: neuroactive ligand-receptor interaction	CHRM2, OPRD1, CHRM3, PRSS1, CHRM1, CHRNA2, CHRM4, CHRNA7, CHRM5, HTR2C, ADRA1D, ADRB2, HTR2A, ADRA1B, NR3C1, ADRA1A, EDNRA, CALCR, DRD1, GABRE, DRD2, DRD5, GABRA2, GABRA1, GABRA6, GABRA5, HTR1A, HTR1B, OPRM1, ADRA2C, F2, GABRG3, ADRA2B, ADRA2A	3.64E-19	34
3	hsa05161: hepatitis B	RB1, CDKN1A, JUN, PCNA, STAT3, FOS, TNF, MMP9, PIK3CG, RELA, CASP9, NFKBIA, CCNA2, IL6, CCND1, CDK4, MYC, CASP3, CDK2, BCL2, BIRC5, AKT1, MAPK1, TP53	3.15E-16	24
4	hsa05219: bladder cancer	RB1, CDKN1A, MMP1, MMP2, MMP9, EGFR, VEGFA, CCND1, CDK4, MYC, ERBB2, MDM2, MAPK1, TP53	1.04E-13	14
5	hsa05215: prostate cancer	RB1, GSK3B, CDKN1A, HSP90AA1, EGFR, PIK3CG, RELA, CASP9, NFKBIA, AR, CCND1, ERBB2, CDK2, MDM2, BCL2, AKT1, MAPK1, TP53	1.17E-13	18
6	hsa04151: PI3K-Akt signaling pathway	CHRM2, GSK3B, CDKN1A, CHRM1, ITGB3, RELA, EGFR, PIK3CG, CASP9, RXRA, CCND1, MYC, AKT1, MAPK1, MCL1, HSP90AA1, NOS3, INSR, IL2, VEGFA, IL4, IL6, CDK4, CDK2, BCL2, MDM2, MET, TP53, BCL2L1	5.55E-12	29
7	hsa04066: HIF-1 signaling pathway	CDKN1A, EDN1, NOS2, NOS3, INSR, STAT3, EGFR, PIK3CG, RELA, VEGFA, IL6, IFNG, ERBB2, BCL2, AKT1, HMOX1, MAPK1	7.13E-12	17
8	hsa05222: small cell lung cancer	RB1, NOS2, PTGS2, PIK3CG, RELA, CASP9, NFKBIA, RXRA, CCND1, CDK4, MYC, CDK2, BCL2, AKT1, TP53, BCL2L1	1.43E-11	16
9	hsa05212: pancreatic cancer	RB1, STAT3, EGFR, PIK3CG, RELA, VEGFA, CASP9, CCND1, CDK4, ERBB2, AKT1, MAPK1, TP53, BCL2L1	6.79E-11	14
10	hsa05210: colorectal cancer	GSK3B, JUN, FOS, PIK3CG, CASP9, CCND1, MYC, CASP3, BCL2, BIRC5, AKT1, MAPK1, TP53	5.73E-10	13
11	hsa04024: cAMP signaling pathway	CHRM2, JUN, CHRM1, HTR1A, HTR1B, FOS, ADRB2, ADCY8, PIK3CG, RELA, NFKBIA, EDNRA, CAMK4, PDE3A, AKT1, MAPK1, DRD1, DRD2, PRKACA, DRD5	1.36E-09	20
12	hsa04915: estrogen signaling pathway	JUN, HSP90AA1, NOS3, MMP2, FOS, OPRM1, ADCY8, ESR1, MMP9, EGFR, PIK3CG, ESR2, AKT1, MAPK1, PRKACA	1.53E-09	15
13	hsa04725: cholinergic synapse	CHRM2, ACHE, CHRM3, CHRM1, CHRM4, CHRNA7, CHRM5, FOS, ADCY8, PIK3CG, CAMK4, BCL2, AKT1, MAPK1, PRKACA	7.09E-09	15
14	hsa04068: foxo signaling pathway	IL10, CDKN1A, INSR, STAT3, SLC2A4, MAPK14, EGFR, PIK3CG, IL6, CCNB1, CCND1, CDK2, MDM2, AKT1, MAPK1	8.18E-08	15
15	hsa04931: insulin resistance	NFKBIA, GSK3B, PTPN1, IL6, NOS3, INSR, STAT3, AKT1, SLC2A4, TNF, RELA, PIK3CG	2.80E-06	12
16	hsa04726: serotonergic synapse	CASP3, HTR1A, HTR1B, MAPK1, HTR2C, HTR3A, HTR2A, PRKACA, PTGS2, SLC6A4, PTGS1	2.42E-05	11
17	hsa05216: thyroid cancer	RXRA, CCND1, MYC, MAPK1, PPARG, TP53	1.36E-04	6
18	hsa04932: nonalcoholic fatty liver disease	GSK3B, IL6, CASP7, JUN, RXRA, CASP3, INSR, AKT1, TNF, RELA, PIK3CG	3.24E-04	11
19	hsa04152: AMPK signaling pathway	CCNA2, CCND1, FASN, INSR, AKT1, PPARG, SLC2A4, ADRA1A, PIK3CG	0.001461352	9
20	hsa05204: chemical carcinogenesis	CHRNA7, GSTP1, CYP1A2, CYP1A1, CYP3A4, PTGS2	0.013489355	7

**Table 4:** Docking results for the core components of *Salvia miltiorrhiza* and key target proteins.

	Affinity (kcal/mol)						
Target	Original ligands	Isocryptotan-shinone	Dihydrosalvian-olone	Salvia miltiorrhiza new quinone D	Tanshinone IIA	Salviol ketone	Luteolin
PTGS2 (5ikv)	-9.08	-9.82	-9.23	-10.54	-10.06	-9.26	-8.25
OPRM1 (6ddf)	-2.47	-7.81	-8.05	-7.74	-8.73	-8.65	-7.38
NCOA1 (5nma)	-9.98	-9.40	-8.51	-9.36	-9.50	-8.26	-7.42
CHRM1 (6oij)	-5.24	-8.42	-7.24	-9.06	-8.05	-7.55	-7.00

## Data Availability

The data used to support the findings of this study are all included within the article.
